RETRACTED

# Study on the Global Stability for a Generalized SEIR Epidemic Model

**DOI:** 10.1155/2022/8215214

**Published:** 2022-08-08

**Authors:** Chunrong Xue

**Affiliations:** School of Mathematics and Statistics, Weinan Normal University, Weinan, Shaanxi 714000, China

## Abstract

In the current study, a generalized SEIR epidemic model is studied. The generalized fractional-order SEIR model (susceptible-infected-recovered (SIR) epidemic) model differentiated the population into susceptible population, exposure population, infected population, and rehabilitation population and has fundamental mentoring importance for the forecast of the probable outburst of infectious ailments. The fundamental duplicated quantity *R*_0_ is inferred. When *R*_0_ < 1, the disease-free equilibrium (DFE) is particular and tending towards stability. When *R*_0_ > 1, the endemic equilibrium is sole. In addition, certain circumstances are set up to make sure the local progressive stability of disease-free and endemic equilibrium. Considering the influence of the individual behavior, a broader SEIR epidemic model is raised, which classified the population into susceptible, exposure, infected, and rehabilitation. What is more, the basic reproduction number, that regulates whether the infection will die out or not, is obtained by the spectral radius of the next-generation matrix; moreover, the global stability of DFE and endemic equilibrium are analyzed by a geometry method.

## 1. Introduction

Nowadays, some infectious diseases are still aimed at large populations [1, 2]. They are regarded as the potential causes of death, particularly in numerous developing countries [3, 4]. As a result of this, mathematical modeling in epidemiology plays a more and more important role in public health research [5, 6]. This academic subject facilitates interpreting the studies in epidemiological phenomena and catch the distinctive elements that could result in a serious epidemic or even to a hazardous pandemic in the world [7, 8]. The established susceptible-infected-recovered (SIR) epidemic model was firstly described by Kermackin 1991 [9].The infection latency often needs a long-time range [7] In the meantime, an incubated individual is still latent but hasn't contagious [10]. Consequently, another type of exposed individuals might be supplemented to SIR and the novel epidemic model SEIR was introduced by Ricardo [11]. This SEIR model with treatment and offeredcertain adequate conditions to certify the local stability of equilibrium points. Additionally, epidemiological studies have exposed that mutation leads to more and more unaffected viruses offering the emergence of numerous new damaging epidemics or even new hazardous pandemics [12]. The laws of disease spreading should be urgently investigated because of infectious diseases bring disaster to human health and might provide a theoretical basis for the infection prevention and control [13]. Due to infectious disease existing certain latency before its breaking out, the SEIR epidemic model was researched in a latent period. As described in the study [14], Zhang, Li, and Ma et al. analyzed an SEIR epidemic model with the immigration of different compartments and adequate contact rates and proved the overall stability of the system by variable transformation. In addition, Meng, Chen, and Song introduced the delayed SEIR epidemic model with perpendicular propagation and pulsed vaccination [15].They considered the infection-free periodic solution, which was globally attractive under some appropriate conditions; furthermore, time delay, pulse vaccination and vertical transmission brought obvious efforts to the dynamics of the model. The previous research [16] contained random agitations into SIR and SEIR epidemic models with saturated incidence and set that the solution under some conditions had ergodic property by utilizing the stochastic Lyapunov function. Li and Chen discussed an age structured SEIR epidemic model with vertically and horizontally transformation. They established the threshold of endemic existence and showed threshold parameters usually computable in [17]. Chen et al. [18] investigated an SEIR epidemic Model with a non-monotone incidence, then obtained the global stability. It's worth repeating: the morbidity provides further data about the disease broadcast. Therefore, the overall incidence characteristic has as aim of denoting a big collection of infection incidence rate. Meng group, Michael Y. Li, and Ke Wang in [19] considered an SEIR epidemic model for the dynamic transmit of communicable disease that propagate in population by connecting to hosts and analyzed a geometric method to global stability. A great deal of processes of mutation was detected in a large number of communicable diseases. Due to this reason, the multi-strain SEIR epidemic model is a critical tool for investigating a number of communicable diseases that comprise a lengthy incubation period and also diverse infection strains. The correlation of learning multi-strain models is finding out the diverse situations allowing all operating strains to coexist. The global dynamics of the SEIR model is the focus of numerous explorations by studying bilinear or nonlinear incidence. In the current study, a comprehensive SEIR epidemic model is studied, and the threshold is obtained. By the method of geometric approach, global stability of disease-free equilibrium (DFE) and endemic equilibrium are analyzed; furthermore, the infection will die away if *R*_0_ < 1, or become endemic if *R*_0_ > 1.

RETRACTED

## 2. Preliminaries and Model Derivation

The incidence provides further evidence about the spread of the disease [20] Therefore, the goal of the general incidence rate function is to characterize the incidence rate of a large group of infections. Consequently, the aim of this study is to summarize the earlier models by thinking over a SEIR model with general prevalence rate. Therefore, this current study would be carried out on the subsequent comprehensive SEIR epidemic model:

(1) $$\begin{array}{c} \left\{\begin{array}{c} \frac{\text{d}S}{\text{d}t}=A-f\left(S,I\right)-dS,\\ \frac{\text{d}E}{\text{d}t}=f\left(S,I\right)-\varepsilon E-dE,\\ \frac{\text{d}I}{\text{d}t}=\varepsilon E-\delta I-dI,\\ \frac{\text{d}R}{\text{d}t}=\delta I-dR, \end{array}\right. \end{array}$$

where (S)is the numbers of susceptible population; (E)is the numbers of each latent individual's class;(I) denotes the amount of communicable population;(R) is the amount of deleted population; With regard to the issues coping with population dynamics, all the variables might be positive. We would suppose firstly that all the model indicators are positive. The paraments A is positive constant, which represents the birth rate of the population. The paraments d is positive invariable too, which represents the death rate of the population. The non-negative constant *ε* describes the transfer rates from exposed to infected, and the non-negative constant *δ* describes the transmission rates from infection to recovery. The function *f* (S, I) represents the ratio of new infection and is expected to be sufficiently smooth to ensure the existence and uniqueness of solution to the system (1) with non-negative initial situations. By the functional framework of basic theory of differential equations, we verify that there is a particular local solution to the issues. To verify the positive results, we would demonstrate that any settlement beginning from positive orthant. To meet biological sense, the function f (S, I) is assumed to fulfill the conditions as below for all S ≥ 0, I ≥ 0:

- *f*(0,0)=*f*(*S*, 0)=*f*(0, *I*)=0,
- *f*(*S*, *I*) > 0 for *S* > 0,  *I* > 0,
- *∂f*(*S*, *I*)/*∂S* ≥ 0, (*∂f*(*S*, *I*)/*∂I*) > 0,
- *I*(*∂f*(*S*, *I*)/*∂I*) ≥ *f*(*S*, *I*),
- *I*(*∂f*(*S*, *I*)/*∂I*) − *E*(*∂f*(*S*, *I*)/*∂S*) − *f*(*S*, *I*) > 0.

The total population *N*=*S*+*E*+*I*+*R* satisfies *N*′=*A* − *dN* may vary in time. It is easy to see the population scale *N* converges to (*A*/*d*) without disease, thus we study system (1) in the following feasible region:

(2) $$\begin{array}{c} D=\left\{\left(S,E,I,R\right)\in R_{+}^{4}:S+E+I+R\leq \frac{A}{\text{d}}\right\}. \end{array}$$

Which is a positive invariant set in *R*_+_^4^, represents the border and inner of *D* by *∂D* and *D*° respectively.

RETRACTED

The condition (a) ensures the existence of unique DFE *P*_0_(*A*/d, 0,0,0) ∈ *∂D* for system (1). Setting the right-hand sides of the last three equation to zero, and the sum of the first two equation to zero, it is easy to obtain a particular endemic equilibrium *P*^*∗*^(*S*^*∗*^, *E*^*∗*^, *I*^*∗*^, *R*^*∗*^), where,

(3) $$\begin{array}{c} S^{*}=\frac{A\varepsilon -\left(\text{d}+\varepsilon \right)\left(\text{d}+\delta \right)I^{*}}{\text{d}\varepsilon },\\ E^{*}=\frac{\text{d}+\delta }{\varepsilon }I^{*},\\ R^{*}=\frac{\delta }{\text{d}}I^{*} \end{array}$$

Simultaneously obtained

(4) $$\begin{array}{c} f\left(S^{*},I^{*}\right)=\frac{\left(\text{d}+\varepsilon \right)\left(\text{d}+\delta \right)}{\varepsilon }I^{*},\\ \frac{\partial f}{\partial I}\left(S^{*},I^{*}\right)=\frac{\left(\text{d}+\varepsilon \right)\left(\text{d}+\delta \right)}{\varepsilon }. \end{array}$$

## 3. The Basic Reproduction Number

In this section, the basic reproduction number *R*_0_ is studied. *R*_0_ is clarified as the spectral radius of next-generation matrix in [7], i.e.

In this section we study the fundamental reproduction number *R*_0_, *R*_0_ is expressed as the spectral radius of next-generation matrix in [7], i. e. *R*_0_=*ρ*(*FV*^−1^). In system (1), only *E* and *I* is directly related to epidemic. There followed the way of van den driessche and Watmough, that is

(5) $$\begin{array}{c} \left(\begin{array}{c} \frac{\text{d}E}{\text{d}t}\\ \frac{\text{d}I}{\text{d}t} \end{array}\right)=\left(\begin{array}{c} f\left(S,I\right)\\ 0 \end{array}\right)-\left(\begin{array}{c} \left(\text{d}+\varepsilon \right)E\\ -\varepsilon E+\left(d+\delta \right)I \end{array}\right),\\ F=\left(\begin{array}{cc} 0 & \frac{\partial f}{\partial I}\left(\frac{A}{\text{d}},0\right)\\ 0 & 0 \end{array}\right),\\ V=\left(\begin{array}{cc} d+\varepsilon & 0\\ -\varepsilon & d+\delta \end{array}\right), \end{array}$$

then $V^{-1}=\left(1/\left(d+\varepsilon \right)\left(d+\delta \right)\right)\left(\begin{array}{cc} d+\delta & 0\\ \varepsilon & d+\varepsilon \end{array}\right)$

The next-generation matrix is

(6) $$\begin{array}{c} FV^{-1}=\frac{1}{\left(\text{d}+\varepsilon \right)\left(\text{d}+\delta \right)}\left(\begin{array}{cc} \varepsilon \frac{\partial f}{\partial I}\left(\frac{A}{\text{d}},0\right) & \left(d+\varepsilon \right)\frac{\partial f}{\partial I}\left(\frac{A}{\text{d}},0\right)\\ 0 & 0 \end{array}\right). \end{array}$$

Hence the fundamental reproduction number as,

(7) $$\begin{array}{c} R_{0}=\frac{\varepsilon }{\left(\text{d}+\varepsilon \right)\left(\text{d}+\delta \right)}\frac{\partial f}{\partial I}\left(\frac{A}{\text{d}},0\right). \end{array}$$

RETRACTED

## 4. Global Stabilities of Disease-free Equilibrium (DFE)

The disease-free equilibrium (DFE) is characterized by the demising of the infecting, and the sickness could not attack the individuals. The DFE first nonzero component is determined by the infant natality and mortality of the predisposed population and does not rely on the morbidity functional indicators. The infection disappeared, the susceptibility gets their greatest numerical, and the rest of variables eliminate. In this paragraph, concentration might be concentrated to the statistical stability of this DFE. In fact, we could suppose the stability of DFE when the fundamental reproduction quantity is less than the unified value. This makes us to seek for the proper model indicators to inspect statistically the steadiness of the original stable status.

By the framework of van den Driessche and Watmough [21], we immediately obtained the following local asymptotical stability of DFE:

**Theorem 1 .**

Allow *R*_0_ be defined in (7), the unique DFE of system (1) is local asymptotical stability provided that *R*_0_ < 1 and unsteady provided that *R*_0_ > 1.

To explore the global stability of DFE, the following result explained in [22]is needed:

**Lemma 1 .**

Take into account a model expressed in a form

(8) $$\begin{array}{c} \left\{\begin{array}{c} \frac{dX_{1}}{dt}=F\left(X_{1},X_{2}\right)\\ \frac{dX_{2}}{dt}=G\left(X_{1},X_{2}\right),G\left(X_{1},0\right)=0 \end{array}\right., \end{array}$$

where *X*_1_ ∈ *R*^*m*^ represents the amount of population without infection and *X*_2_ ∈ *R*^*m*^ represents the sum of infected population containing potential, infectious, etc; *X*_0_=(*X*_1_^*∗*^, 0) indicates the DFE of system (8).

Also suppose the conditions (H1) and (H2) as following:

(H1) For d*X*_1_/d*t*=*F*(*X*_1_, 0), *X*_1_^*∗*^ is global asymptotical stability.

(H2) $G\left(X_{1},X_{2}\right)=AX_{2}-\hat{G}\left(X_{1},X_{2}\right)$, $\hat{G}\left(X_{1},X_{2}\right)\geq 0$ for (*X*_1_, *X*_2_) ∈ Ω, the Jacobian matrix *A*=(*∂G*/*∂X*_2_)(*X*_1_^*∗*^, 0) is an M-matrix and Ω is the feasible region.

Then the DFE *X*_0_=(*X*_1_^*∗*^, 0) is global asymptotical stability if *R*_0_ < 1.

**Theorem 2 .**

The DFE of system (1) is global asymptotical stability if *R*_0_ < 1.

**Proof**

In system (1), permit *X*_1_=(*S*, *R*)^*T*^, *X*_2_=(*E*, *I*)^*T*^, the uninfected model is

(9) $$\begin{array}{c} \left(\begin{array}{c} \frac{\text{d}S}{\text{d}t}\\ \frac{\text{d}R}{\text{d}t} \end{array}\right)=F\left(X_{1},X_{2}\right)=\left(\begin{array}{c} A-f\left(S,I\right)-dS\\ \delta I-dR \end{array}\right), \end{array}$$

the infected model is

(10) $$\begin{array}{c} \left(\begin{array}{c} \frac{\text{d}E}{\text{d}t}\\ \frac{\text{d}I}{\text{d}t} \end{array}\right)=G\left(X_{1},X_{2}\right)=\left(\begin{array}{c} f\left(S,I\right)-\left(d+\varepsilon \right)E\\ \varepsilon E-\left(d+\delta \right)I \end{array}\right). \end{array}$$

and *G*(*X*_1_, 0)=0.

RETRACTED

Next requireto verify the conditions (H1) and (H2).

When *X*_2_=0, i.e. *E*=*I*=0, the model (9) is

(11) $$\begin{array}{c} \left(\begin{array}{c} \frac{\text{d}S}{\text{d}t}\\ \frac{\text{d}R}{\text{d}t} \end{array}\right)=\left(\begin{array}{c} A-dS\\ -dR \end{array}\right). \end{array}$$

And the solution of system (11) is *S*(*t*)=*A*/d − (*S*(0) − (*A*/d))*e*^−*dt*^, *R*(*t*)=*R*(0)*e*^−*dt*^.

It is easy to see *S*(*t*)⟶*A*/d, *R*(*t*)⟶0, as *t*⟶+*∞*. Hence *X*_1_^*∗*^(*A*/d, 0) is global asymptotical stability. The condition (H1) is verified.

(12) $$\begin{array}{c} G\left(X_{1},X_{2}\right)=\frac{\partial G}{\partial X_{2}}\left(X_{1}^{*},0\right)X_{2}-\hat{G}\left(X_{1},X_{2}\right)\\ =\left(\begin{array}{cc} -\left(\text{d}+\varepsilon \right) & \frac{\partial f}{\partial I}\left(\frac{A}{\text{d}},0\right)\\ \varepsilon & -\left(\text{d}+\delta \right) \end{array}\right)\left(\begin{array}{c} E\\ I \end{array}\right)-\left(\begin{array}{c} I\frac{\partial f}{\partial I}\left(\frac{A}{\text{d}},0\right)-f\left(S,I\right)\\ 0 \end{array}\right), \end{array}$$

obviously *A*=(*∂G*/*∂X*_2_)(*X*_1_^*∗*^, 0) is an M-matrix. According to assumption (d) we obtain $\hat{G}\left(X_{1},X_{2}\right)\geq 0$. The condition (H2) is verified.

According to Lemma 1, The DFE *P*_0_(*A*/d, 0,0,0) of system (1) is global asymptotical stability if *R*_0_ < 1.

## 5. Global stabilities of endemic equilibrium

**Theorem 3 .**

There exists a unique positive endemic equilibrium for system (1) if *R*_0_ > 1, and no positive endemic equilibrium if *R*_0_ < 1.

Let *F*(*I*)=*f*(*S*^*∗*^, *I*)/*I*=*f*(*Aε* − (d+*ε*)(d+*δ*), *I*/d*ε*, *I*)/*I*, *y*=(d+*ε*)(d+*δ*)/*ε*. Let y=F(I)

(13) $$\begin{array}{c} f\left(\frac{A\varepsilon -\left(\text{d}+\varepsilon \right)\left(\text{d}+\delta \right)I}{\text{d}\varepsilon },I\right)=\frac{\left(\text{d}+\varepsilon \right)\left(\text{d}+\delta \right)}{\varepsilon }. \end{array}$$

It is clearly to see *F*(*I*)=0 at *I*=(*Aε*/(d+*ε*)(d+*δ*)), then

(14) $$\begin{array}{c} F\left(I\right)<\frac{\left(\text{d}+\varepsilon \right)\left(\text{d}+\delta \right)}{\varepsilon }. \end{array}$$

with the help of inequality (d)

(15) $$\begin{array}{c} \underset{I⟶0^{+}}{\text{lim}}F\left(I\right)=\underset{I⟶0^{+}}{\text{lim}}\frac{f\left(A/\text{d},0\right)}{I}=\frac{\partial f}{\partial I}\left(\frac{A}{\text{d}},0\right)>\frac{\left(\text{d}+\varepsilon \right)\left(\text{d}+\delta \right)}{\varepsilon }. \end{array}$$

The equation y =F(I) has unique solution if and only if *∂f*/*∂I*(*A*/d, 0) > ((d+*ε*)(d+*δ*)/*ε*), then *ε∂f*/*∂I*(*A*/d, 0)/(d+*ε*)(d+*δ*) > 1 , namely *R*_0_ > 1.

RETRACTED

Clearly *R*_0_ > 1, there is a unique positive endemic equilibrium for system (1), and no positive endemic equilibrium for *R*_0_ < 1.

**Theorem 4 .**

The unique positive endemic equilibrium of system (1) is local asymptotical stability provided that *R*_0_ > 1.

Proof To study the local asymptotical stability, the equivalent system of (1) is researched

(16) $$\begin{array}{c} \left\{\begin{array}{c} \frac{dS}{dt}=A-f\left(S,I\right)-dS\\ \frac{dE}{dt}=f\left(S,I\right)-\left(d+\varepsilon \right)E\\ \frac{dI}{dt}=\varepsilon E-\left(d+\delta \right)I. \end{array}\right. \end{array}$$

The Jacobian matrix of system (16) is

(17) $$\begin{array}{c} J=\left(\begin{array}{c} -\frac{\partial f}{\partial S}\left(S,I\right)-d0-\frac{\partial f}{\partial I}\left(S,I\right)\\ \frac{\partial f}{\partial S}\left(S,I\right)-\left(d+\varepsilon \right)\frac{\partial f}{\partial I}\left(S,I\right)\\ 0\varepsilon -\left(d+\delta \right) \end{array}\right), \end{array}$$

and the characteristic equation at *P*^*∗*^(*S*^*∗*^, *E*^*∗*^, *I*^*∗*^, *R*^*∗*^) is

(18) $$\begin{array}{c} \text{Det}\left(\lambda E-J\right)=\lambda^{3}+a_{1}\lambda^{2}+a_{2}\lambda +a_{3}=0, \end{array}$$

where *a*_1_=3  *d*+*ε*+*δ*+(*∂f*/*∂S*)(*S*^*∗*^, *I*^*∗*^) > 0, *a*_2_=(*∂f*/*∂S*(*S*^*∗*^, *I*^*∗*^)+*d*)(2  *d*+*ε*+*δ*) > 0,

(19) $$\begin{array}{c} a_{3}=\varepsilon \frac{\partial f}{\partial I}\left(S^{*},I^{*}\right)\frac{\partial f}{\partial S}\left(S^{*},I^{*}\right)>0. \end{array}$$

In order to prove all roots, have negative real parts, using (4) and obtain *a*_1_ > *d*+*ε*, *a*_2_ > *∂f*/*∂S*(*S*^*∗*^, *I*^*∗*^)(*d*+*δ*), *a*_3_=(*d*+*ε*)(*d*+*δ*)*∂f*/*∂S*(*S*^*∗*^, *I*^*∗*^), therefore *a*_1_*a*_2_ − *a*_3_ > 0.

According to Routh-Hurwitz theory the unique positive endemic equilibrium of system (1) is local asymptotical stability provided that *R*_0_ > 1.

**Theorem 5 .**

The unique positive endemic equilibrium of system (1) is global asymptotical stability provided that *R*_0_ > 1.

Proof In line with Theorem 1 the unique DFE of system (1) is unstable provided that *R*_0_ > 1, and *P*_0_(*A*/d, 0,0,0) ∈ *∂D*, then system (1) is uniform persistence [23], i.e. ∃*c* > 0, $\underset{t⟶\infty }{\text{lim}}\text{inf}\left\{S\left(t\right),E\left(t\right),I\left(t\right)\right\}>c$. Uniform persistence implies the presence of compact subsets *K* ⊂ *D*. It is easy to see system (1) satisfies the conditions in [24].

RETRACTED

Next, we only need to prove the Bendixson criterion *q* < 0.

The Jacobian matrix of system (16) is (17), and the associated second compound matrix is,

(20) $$\begin{array}{c} J^{\left[2\right]}=\left(\begin{array}{c} -\frac{\partial f}{\partial S}\left(S,I\right)-\left(2\;d+\varepsilon \right)\frac{\partial f}{\partial I}\left(S,I\right)\frac{\partial f}{\partial I}\left(S,I\right)\\ \varepsilon -\frac{\partial f}{\partial S}\left(S,I\right)-\left(2\;d+\delta \right)0\\ 0\frac{\partial f}{\partial S}\left(S,I\right)-\left(2\;d+\varepsilon +\delta \right) \end{array}\right). \end{array}$$

Let the matrix function *P*(*S*, *E*, *I*)=diag(1, *E*/*I*, *E*/*I*), then

*P*_*f*_ *P* ^−1^=diag(0, (*E*′/*E*) − (*I*′/*I*), (*E*′/*E*) − (*I*′/*I*)), matrix *B*=*P*_*f*_*P*^−1^+*PJ*^[2]^*P*^−1^ can be written in the form $B=\left(\begin{array}{cc} B_{11} & B_{12}\\ B_{21} & B_{22} \end{array}\right)$where *B*_11_=−(2  *d*+*ε*) − *∂f*/*∂S*(*S*, *I*), *B*_12_=[*∂f*/*∂I*(*S*, *I*)*I*/*E*, *∂f*/*∂I*(*S*, *I*)*I*/*E*], *B*_21_=[*ε*(*E*/*I*), 0]^*T*^,

(21) $$\begin{array}{c} B_{22}=\left(\begin{array}{c} \frac{E^{\prime }}{E}-\frac{I^{\prime }}{I}-\left(2\;d+\delta \right)-\frac{\partial f}{\partial S}\left(S,I\right)0\\ \frac{\partial f}{\partial S}\left(S,I\right)\frac{E^{\prime }}{E}-\frac{I^{\prime }}{I}-\left(2\;d+\varepsilon +\delta \right) \end{array}\right). \end{array}$$

We define a norm ‖(*u*, *v*, *w*)‖=max{|*u*|, |*v*+*w*|} for any vector (*u*, *v*, *w*) in *R*^3^, and *μ*(*B*) denote the Lozinskil measure with respect to this norm. Using the valuation method in [25] we have *μ*(*B*) ≤ sup(*g*_1_, *g*_2_), with *g*_1_=*μ*_1_(*B*_11_)+|*B*_12_|,

*g*_2_=|*B*_21_|+*μ*_1_(*B*_22_). |*B*_12_|, |*B*_21_| are the matrix norm about *l*_1_ vector norm, *μ*_1_ is Lozinskil measure about *l*_1_ norm. For example, $\left|A\right|=\underset{1\leq k\leq n}{\text{max}}\sum_{i=1}^{n}\left|a_{ik}\right|,$$\mu_{1}\left(A\right)=\underset{1\leq k\leq n}{\text{max}}\left(a_{kk}+\sum_{i=1,i\neq k}^{n}\left|a_{ik}\right|\right)$ for any matrix *A*=(*a*_*ij*_)_*n*×*n*_, then

(22) μB111=−2d+ε−∂f∂SS,I,B12=∂f∂IS,IIE,B21=εEI,μB221=E′E−I′I−2d+δ.

Hence

(23) $$\begin{array}{c} g_{1}=-\left(2\;d+\varepsilon \right)-\frac{\partial f}{\partial S}\left(S,I\right)+\frac{\partial f}{\partial I}\left(S,I\right)\frac{I}{E},\\ g_{2}=\varepsilon \frac{E}{I}+\frac{E^{\prime }}{E}-\frac{I^{\prime }}{I}-\left(2\;d+\delta \right). \end{array}$$

From system (16), we obtain *I*′/*I*=*ε*(*E*/*I*) − (*d*+*δ*) and−(*d*+*ε*)=(*E*′/*E*) − (*f*(*S*, *I*)/*E*),then *g*_2_=*E*′/*E* − *d* and *g*_1_=((*E*′/*E*) − (*f*(*S*, *I*)/*E*) − *d* − (*∂f*/*∂S*)(*S*, *I*)+(*∂f*/*∂I*)(*S*, *I*)(*I*/*E*)), by assumption (e), *g*_1_=((*E*′/*E*) − *d* − (*∂f*/*∂S*)(*S*, *I*) < (*E*′/*E*) − *d*), then *μ*(*B*) ≤ sup(*g*_1_, *g*_2_)=(*E*′/*E*) − *d*.

Since system (1) is uniform persistence, there is *ξ* > 0, *T* > 0 so that when *t* > *T* , *E*(*t*) > *ξ*, *I*(*t*) > *ξ* for all (*S*(0), *E*(0), *I*(0)) ∈ *K*, we have 1/*t*ln(*E*(*t*)/*E*(0)) < d/2, then 1/*t*∫_0_^*t*^*μ*(*B*)d*s* ≤ (1/*t*)ln*E*(*t*)/*E*(0) − *d* < −(d/2), namely

$q=\underset{t⟶\infty }{\text{lim}}\text{sup}\underset{x_{0}\in K}{\text{sup}}$ 1/*t*∫_0_^*t*^*μ*(*s*, *x*_0_)d*s* < −(d/2) < 0, thus, the associated second compound matrix is local asymptotical stability, verified the proof.

RETRACTED

## 6. Discussion and conclusion

It is well described that the spreading of a contagious illness implicates disease-related elements including infectious mediator, route of broadcast, latent period, infectious stage, susceptivity, and resistance [26]. Infectious disease model defining a spread mediators in an enclosed population and containing susceptible (S), infectives (I), and recovers (R) were introduced by Kermack in 1927. According to the Kermack model, diverse epidemic models have been advanced in current periods, such as SIR, SIS, SEIR models [27]. Functional form of the incidence rate plays a critical role in of epidemic model. Several previous studies highlight that the route of disease transmission might have a nonlinear incidence ratio [28]. To explore the effect of the non-linearity, Korobeinikov take into account diversified models with the incidence and set up Lyapunov functions that make them to create global properties for SEIR model. Thereafter, Korobeinikov proven global properties for multiple epidemic models with incidence of a more commonformula [29].

In the current study, we have explored the global stability of the generalized SEIR model with quantitative overview of the complex analysis and certain qualitative characteristics of the SEIR model have been discussed. This model included some compartments, namely the susceptible, exposing individuals, infecting individuals, and the removal individuals. We have created the existence, positivity and boundedness of settlement which ensure the well-formedness of the SEIR model. To validate our distinctive results theoretically, numerical simulation is carried out. It is measured that the model with extensive association capabilities contains many typical correlation features, which could better understand the equilibrium stability. The long-term forecast desires to amend the model properly based on the alteration of strategic and medical aspects. We might talk about this in the future work.

RETRACTED

## Data Availability

The datasets used and analyzed during the current study are available from the corresponding author on reasonable request.
